RETRACTED

# *Camellia sinensis* methanolic leaves extract: Phytochemical analysis and anticancer activity against human liver cancer cells

**DOI:** 10.1371/journal.pone.0309795

**Published:** 2024-11-14

**Authors:** Demiana H. Hanna, Ahlam K. Al-Atmani, Aljazi Abdullah AlRashidi, E. El. Shafee

**Affiliations:** 1 Faculty of Science, Department of Chemistry, Cairo University, Giza, Egypt; 2 Faculty of Science, Department of Chemistry, University of Hail, Hail, Saudi Arabia; University of Ibadan Faculty of Science, NIGERIA

## Abstract

**Background:**

The study’s primary goal is to ascertain whether there is a relationship between the processed green tea methanolic extract’s (GTME) phytochemical components and its potential effectiveness against human liver cancer cells. The GTME’s phytochemical composition was identified using gas chromatography-mass spectrometry, and the extract’s capacity to lower cellular proliferation and cause apoptosis in HepG2 cancerous liver cell lines was checked.

**Results:**

The findings of the gas chromatography-mass chromatogram showed that GTME included bioactive antioxidants and anticancer substances. Additionally, utilizing the MTT, comet assay, and acridine assay, GTME revealed a selective cytotoxic impact with a significant IC_50_ value (27.3 µg/ml) on HepG2 cells without any harmful effects on WI-38 healthy cells. Also, compared to untreated cells, the extract-treated HepG2 cells had an upsurge in the proportion of cells that have undergone apoptosis and displayed a comet nucleus, which is a sign of DNA damage. In addition, HepG2 cells treated with GTME revealed a stop in the G1 phase and sub-G1 apoptotic cells (37.32%) in a flow cytometry analysis. Furthermore, reactive oxygen species were shown to be responsible for HepG2 apoptosis, and the tested extract significantly reduced their levels in the treated cells. Lastly, compared to untreated cells in treated HepG2 cells, GTME significantly changed protein expression levels linked with cell cycle arrest in the G1 phase and apoptosis.

**Conclusion:**

These findings provided information about the processes through which the GTME inhibited the growth of HepG2. Therefore, it has potential as an effective natural therapy for the treatment of human liver cancer. However, to validate these findings, animal models must be used for *in vivo* studies.

## Background

Liver cancer ranks fourth globally in terms of cancer-related deaths, following stomach, lung, and colorectal cancer **[1].** It is also the sixth—most commonly diagnosed malignancy. With an incidence-to-mortality ratio that is close to one and the majority of cases being discovered at advanced stages, liver cancer is a very deadly tumor **[2]**. Hepatocellular carcinoma (HCC) is a major global health concern that accounts for approximately 75–85% of primary liver malignancies **[3]**. Reactive oxygen species (ROS)-induced hepatocellular damage and the development of chronic inflammation linked to hepatocarcinogenesis occur prior to the induction of HCC **[4].** The HCC has been defeated by adjuvant treatments such as doxorubicin, interferon alpha, and 5-FU; or tumor necrosis factor and melphalan; or cisplatin, epirubicin, and 5-FU **[5]**. Nevertheless, the primary issue with chemotherapy for HCC treatment is the cancer resistance mechanism, which results from a decrease in apoptotic proteins and an up-regulation of the multi-drug resistance protein **[6]**. Consequently, in order to successfully treat cancer, apoptosis induction must be induced, and this requires more potent chemotherapy **[7]**.

RETRACTED

As a result of the chemotherapeutic issues, including hepatotoxicity, recurrence, drug resistance, and other undesirable effects, researchers are now forced to look at alternative therapy choices with fewer side effects and higher therapeutic efficacy. Moreover, the anticarcinogenic medicines currently being studied in human cancer research trials have significant drawbacks, including their high cost, the inevitable long-term subcutaneous or intravenous treatment, and frequently their propensity to kill some healthy cells along with cancer cells. So, much research has been conducted to find potential natural cancer treatments that could be beneficial in the treatment and prevention of malignancies.

Natural remedies derived from plants can be used to cure a variety of illnesses without the harmful side effects linked to synthetic medicines **[8,9]**. In the past few decades, natural compounds have been considered to be important sources of potential chemotherapeutic medicines. There has been a lot of interest in the potential of bioactive substances found in natural products for preventing cancer. Plants have long been used to cure various cancer cells **[10]**. Numerous naturally occurring substances and plant extracts have shown antioxidant and anticancer potential in a range of bioassay systems and animal models relevant to human diseases, according to experimental research **[11]**. Phenolic chemical constituents have been linked to the antioxidant and anti-cancer properties of extracts derived from medicinal plants and herbs. Flavonoids, tannins, quinones, coumarins, lignans, phenolic acids, stilbenes, and curcuminoids were the main categories of phenolic chemicals **[12]**.

Green tea, one of the most important natural plants, is derived from the leaves of the natural species Camellia sinensis, and it is well recognized as one of the most widely consumed beverages on a global scale. About 15–20% of green tea’s protein is composed of amino acids, including tyrosine, threonine, 5-N-ethylglutamine, glutamic acid, aspartic acid, and others. Additionally, it has traces of metals like magnesium and carbohydrates such as glucose, cellulose, and sucrose **[13]**. Consumers are also benefiting from its reported antioxidant, anti-inflammatory, and antibacterial qualities **[14]**. The most abundant and effective class of tea components are called polyphenols, and they comprise the cancer chemopreventive potentials of representative polyphenols in green tea (caffeic acid, CA; gallic acid, GA; catechin, C; epicatechin, EC; gallocatechin, GC; catechin gallate, CG; gallocatechin gallate, GCG; epicatechin gallate, ECG; epigallocatechin, EGC; and epigallocatechin gallate, EGCG) **[15]**. Cancer development, propagation, and progression are all inhibited by the chemopreventive and chemotherapeutic effects of green tea polyphenols **[16]**. Antioxidant action, protection against DNA damage, suppression of proteasome activity, activation of apoptosis, modulation of the cell cycle and proliferation, and avoidance of tumor-promoting events are just some of the biological effects attributed to green tea polyphenols **[17,18]**.

RETRACTED

Previous research has demonstrated the effectiveness of methanol green tea extract in suppressing various cancer cells, such as human cervical cancer cells **[19]** and renal carcinoma cells **[20]**. Nevertheless, research on the harmful effects of methanol green tea extract on human liver cancer cells has not yet been conducted. Therefore, the purpose of this work is to quantify the potential effect of the methanolic green leaf extract on inhibiting the growth and dissemination of HepG2 liver malignant cells and elucidating the various routes involved in the potential activation of apoptosis.

## Methods

### Standards and reagents

Methanol (CAT. No. 322415), DMSO (CAT. No. 5.89569), MTT (CAT. No. M5655), and Minimum Essential Medium (CAT. No. M0268), PBS (CAT. No. P4417), formaldehyde (CAT. No. 252549), Gallic acid (CAT. No. G7384), Quercetin (CAT. No. Q4951), Tannic Acid (CAT. No. 403040), Folin Phenol reagent (CAT. No. F9252), and sodium carbonate solution (CAT. No. 223530) were purchased from Sigma-Aldrich, Saint Louis, USA.

### Plant collection, identification and processing

The leaves and buds of Camellia sinensis, a member of the Theaceae family, were harvested at El-Orman Garden in Giza, Egypt, amid the flowering stage. The taxonomist Mrs. Tressa Labib of El-Orman Garden in Giza, Egypt, graciously identified the plant samples. Voucher specimens (voucher No. CS-322) were placed in the National Research Center’s herbarium in Cairo. The leaves were obtained, repeatedly cleaned with distilled water, evaporated under free airing at temperatures between 35 and 43°C, crushed in a mortar, and then stored at 20°C until needed.

RETRACTED

### Preparation of hydromethanolic extract of green tea leaves

Green tea hydromethanolic extract (GTME) from *Camellia sinensis* leaves was prepared as previously stated **[21]**. An extract-containing solvent was submerged in a solution of 400 g of finely ground green tea leaves for 72 h while being constantly stirred in an equation of 80 methanol to 20 distilled water. After that, the combination was filtered to remove the solvent from the chopped leaves. A rotary evaporator was subsequently utilized to concentrate the end-product solvent three times. After being lyophilized in a freeze-dryer and hardening for 48 h, the extract eventually took the form of a dried green tea hydromethanolic extract (GTME), which was retained at 4°C before usage.

### Quantitative screening of phytochemicals

Using conventional techniques, the initial screening tests for phytochemicals were conducted to determine the valuable components:

### Evaluation of the total phenol content

The total amount of phenols in the green leaf extract was determined using the Folin–Ciocalteau technique and gallic acid (GAE), a standard phenolic component **[21]**. A concentration of one milligram per milliliter was used to prepare the GAE stock solution, and one milligram per milliliter was used to prepare the GTME. Additionally, the standard curve was built using six working concentrations of GAE, which ranged from 15.625 to 500 µg/ml. Using methanol as a blank, the optical density of the samples was measured at 765 nm. The total quantity of phenol in the GTME sample was then computed using the GAE calibration curve by applying the following Formula **(1)**:

TPC=CxV/M (1)

where C is the concentration of GAE in mg/ml that was calculated using the calibration curve, V is the amount of the GTME solution in ml, and M is the mass of the extract in g. TPC is the total phenolic content, which is expressed as mg GAE/g of the GTME. The results were shown as the average of three different trials, with each measurement being performed in triplicate.

### Estimation of the total flavonoid content

A colorimetric aluminum chloride test was employed to determine the total quantity of flavonoids in the produced GTME by measuring quercetin (QE), a standard flavonoid component **[22]**. Both the GTME and the QE stock solution were made with a concentration of one milligram per milliliter in methanol. Moreover, the standard curve was created using six working concentrations of QE, which ranged from 15.625 to 500 µg/ml. Using methanol as a blank, the optical density of the samples was measured at 415 nm. The total flavonoid content of the GTME sample was computed by utilizing the QE calibration curve and the following Formula **(2)**:

C=(cxV)/m (2)

where c is the quantity of QE obtained using the calibration curve (measured in mg/ml), V is the extract’s volume (measured in ml), m is the weight of the tested extract (measured in g), and C is the total amount of flavonoid components represented as mg of QE/g of the GTME. The data were presented as the average of three independent trials, and each measurement was completed in triplicate.

RETRACTED

### Estimation of the total tannin content

The Folin and Ciocalteu method **[23]** was used to measure the GTME’s tannin content. Within distinct test tubes, the GTME (0.1 mL) and the standard Tannic Acid (TAE) solution at six distinct concentrations (from 15.625 to 500 µg/ml) were added. Finally, the volume was increased up to 10 mL with distilled water after adding 7.5 mL of distilled water, 0.5 mL of Folin Phenol reagent, and 1 mL of sodium carbonate solution (35%). Following a thorough shaking of the combination and a 30-minute room temperature hold, the absorbance of the mixture was measured at 725 nm using a Shimadzu UV PC-1600 UV-Vis spectrophotometer against a blank. In milligrams of tannic acid equivalents per gram of extract, the GTME’s total tannin concentration was reported.

### Determining the extract’s phytochemical constituents using gas chromatography-mass spectrometry (GC-MS) analysis

Through the process of derivatization via silylation, the compounds in the extract were identified using GC-MS analysis. The GC analysis of non-volatile and thermolabile substances is best performed via silylation. Trimethylsilyl TMS derivatives have more volatile, less polar, and thermotolerant properties in contrast to their parent compounds. Silylation is the process by which a trimethylsilyl group replaces an active hydrogen in–OH,–COOH, = NH,–NH2, or–SH **[24].** Deploying a mass selective detector (5977A) and a 7890B GC apparatus from Agilent Technologies, the GTME’s chromatographic analysis was successfully completed. The sample was silylated for 2 h at 80°C with N, O-bis (trimethylsilyl) trifluoroacetamide (BSTFA) ahead of insertion onto GC-MS. The column was kept at 60°C for 5 min after the specimen was added, and then it was heated to 300°C using a 20°C/min heating ramp with a hold of 5 min. between 50 and 550 atomic mass units (AMUs), with a solvent delay of 3.0 min and electron impact (EI) ionization at a power level of 70 eV. 8.2 psi of pressure as well as a 1 *µ*l injection of helium were utilized as the carrier gas in a capillary column (HP5MS capillary; 30.0 m, 0.25 mm ID, 0.25 m film). The sample contents were then identified with mass fragmentation and the NIST mass spectral search tool for the NIST/EPA/NIH mass spectral library version 2.2.

RETRACTED

### Anticancer properties

#### Preparation and maintenance of cell lines

The American Type Culture Collection acquired cellular HepG2, a human hepatic cancer cell line, and WI-38, a healthy embryonic lung cell line. Minimum Essential Medium (MEM) was used to cultivate these cells, which were enriched with fetal bovine serum and a mixture of two antibiotics, streptomycin (100 mg/ml) and penicillin (100 U/ml), and housed at 37°C in a CO_2_-filled incubator. Trypsinization created monolayer cells, which were then maintained and used in the following experiments by subculturing in culture flasks.

#### MTT-based cytotoxicity assay

To evaluate the effectiveness of the GTME against the HepG2 malignant cells, the MTT assay, which has been discussed previously **[25,26]**, was used. In short, 1×10^4^ HepG2 cells were seeded in each 96-well plate with the growth MEM medium, and the plates were then incubated at 37˚C for the overnight period. Next, HepG2 cells were treated for 24 h at 37°C with a range of extract dosages (6.25–100 µg/ml). These dosages were first dissolved in DMSO and then diluted with cell culture medium to reach the required final test concentration, while the vehicle control (DMSO) concentration was maintained at or below 0.1%. Next, for four hours at 37˚C, 20 μl of MTT solution (5 mg/ml in PBS) was added to the treated and untreated (control) cells. Insoluble formazan crystals, which are a metabolic byproduct of MTT, were ultimately formed and are strongly correlated with cell viability. On top of that, dimethyl sulfoxide was applied to remove the formazan crystals from the cells. With the goal of expressing the outcome of the green tea extract on cell proliferation, the optical density at 570 nm was measured using a microplate reader (Bio-Rad, USA), and the proportion of HepG2 cell viability was evaluated using the formulae shown in **(3)**.


Cellviability=(Abs.oftestedsample—Abs.ofblank)/(Abs.ofcontrol−Abs.ofblank)x100 (3)

The necessary dose of the examined extract was estimated by a dosage agreement curve (IC_50_) for 50% viability suppression over a 24-h incubation period. To find out whether using the green tea extract on tissues that were alive was secure, all steps of the MTT technique at concentrations between 31 and 500 µg/ml of the extract were performed against healthy embryonic lung cells (WI-38).

RETRACTED

#### Annexin V/PI analysis for apoptosis testing

The phosphatidylserine (PS) transit from the center of the plasma membrane to the outer surface of apoptotic cells provides the basis for the annexin V/PI assay. Hence, implementing the aforementioned Annexin V-FITC detection kit I (BD Biosciences), the percentages of cells that underwent necrosis and apoptosis on either of GTME-treated and untreated HepG2 cells for 24 h were determined, as described earlier **[25,27,28]**. In a nutshell, the extract was only administered to the HepG2 cells for 24 h. After being trypsinized, centrifuged, and rinsed with PBS, the extract-treated and untreated HepG2 cells were incorporated into the Annexin V binding buffer (1x) and then subjected to the dyes Annexin V-FITC and propidium iodide. Using a flow cytometer (BD Biosciences), the results are finally presented as the proportion of each preliminary and advanced apoptotic cell that underwent apoptosis.

#### Fluorescence microscopy-based morphological study

Applying the acridine orange/ethidium bromide stain (AO/EB) method, the control and extract-treated SKOV3 cells’ morphological apoptotic nuclear transformations were examined **[29,30]**. In brief, after being subjected to the GTME, HepG2 cells were rinsed with PBS, fixed in formaldehyde for about 20 min, and stained for two min with AO/EB stain. Ultimately, employing fluorescence microscopy (Carl Zeiss), the nuclear patterns of the control and treated HepG2 cells were investigated, and the rates of cell death were issued. The outcomes represented a consensus of the three assessments after each value was evaluated three times. Ultimately, employing fluorescence microscopy (Carl Zeiss), investigating the nuclear morphology of the untreated and treated HepG2 cells, as well as the cell death rates, was done. The results were the average of the three evaluations after each value was evaluated three times.

#### In *vitro* comet assay

The genotoxicity that was induced in HepG2 cells treated with green tea extract was investigated using the comet assay. Under a fluorescence microscope, strands of damaged DNA will separate from healthy cellular DNA during disintegration. This will end up in a structure that resembles a comet tail. The process involves a number of steps, many of which have already been covered **[28,29]**. For example, 100 images of comets with random shapes were taken using a computerized image analysis system for each slide. TriTek Comet ScoreTM software (TriTek Corp., VA, USA) then analyzed these images to determine the comet parameters. The tail DNA and the tail moment, two commonly utilized signs, were built to be used in discovering the data. It is believed that the Olive tail moment (OTM), also known as a tail moment parameter, represents the most exact estimate that has been used to assess DNA damage. The following Eq **(4)** was applied to determine its value., and it depends on DNA mobility and quantity in the tail.


RETRACTED

OTM=quantityoftailmoment×quantityoftailDNAdividedby100 (4)

All of these comet assay phases were carried out with healthy WI-38 cells in addition to HepG2 cells to evaluate the extract’s genotoxicity with regard to healthy tissues.

#### Examining the variant phases of the cell cycle

Using a cell cycle assay, which analyzes the DNA present in the examined cells, cell division phases were determined. Using the previously described flow cytometry kit (Abcam, catalog ab139418) **[25,28]**, through all phases of the cell cycle, the proportions of untreated and extract-treated cells were measured. HepG2 cells were put into a 6-well culture plate, incubated for an overnight period, and then cultured for 24 h. The extract was then administered to these cells for 24 h, then the cells were gathered, trypsinized, and stored in cold ethanol for an overnight period. The propidium iodide mixture was then applied to these cells for 30 min in the dark and at 37°C. The final phase involved using DNA measurement and flow cytometry to calculate the proportion of cells in every stage of the cell cycle. A histogram representing the results was displayed.

#### ELISA method for quantifying reactive oxygen species (ROS)

According to the manufacturer’s instructions, a human ROS ELISA kit (MyBioSource, USA) was employed to calculate the examined green tea extract’s impact on the formation of ROS in HepG2-treated cells **[25,31]**. In brief, trypsinization, centrifugation, and addition of the supernatant to the relevant wells in a 96-well microplate reader that was covered with an anti-ROS antibody were used to separate the control and green tea extract-treated HepG2 cells. The examined plate was then treated with 100 µl of a working solution containing biotinylated recognition Ab (1x). The conjugate avidin horseradish peroxidase (1x) was poured into the clean wells and left to sit for 30 min at 37°C. Additionally, after being rinsed five times, 90µl of the substrate were placed into the plate’s wells and left in the dark for fifteen minutes. The enzyme-substrate reaction required that the tested plate be thoroughly cleaned and dried before applying about 90 µl of the substrate to each well for fifteen minutes at 37°C for the purpose of producing a blue-colored complex. At last, 50 µl of stop solution were added to each well, creating the yellow solution. Yellow’s absorbance at 450 nm has been evaluated with a microplate reader. The ROS level in the extract-treated cells was calculated using the standard curve, which shows standard doses vs. the intensity of the color. All values were evaluated three times, and the results show the average of the three assessments.

RETRACTED

#### Quantitative Real-Time PCR Technique (qRT-PCR)

The following genes’ mRNA expression levels were evaluated to look into potential processes associated with the result of the green tea extract on cell cycle arrest and apoptosis inside the treated HepG2 cancer cells: genes involved in the cell cycle (*P21*, *P27*, *CDK2*, *CDK4*, *Cyclin E*, *and Cyclin D1*) and genes that regulate apoptosis (*Bax*, *Caspase-3*, *and Bcl-2*). In brief, total RNA was isolated using Thermo Fisher Scientific’s RNA purification kit (catalog #K0731) according to the instructions provided by the manufacturer from both untreated and green tea-treated HepG2 cells. Then, with the intent to gauge the ratio of A260/A280, the quantities of the extracted RNA for every tested sample were acquired. Following the manufacturer’s instructions, first-strand cDNA was generated from the received RNA samples using a kit from Thermo Fisher Scientific termed RevertAid (catalog #K1621). Realtime PCR amplification was carried out using the Thermo Fisher Scientific Maxima SYBR Green qPCR kit (catalog #K0221) and particular primers (Invitrogen) for the investigated genes, as illustrated in **Table 1**. The relative quantification (RQ) of the applied genes was computed using a comparative threshold cycle approach in comparison to their varying expression in the untreated samples and normalized to a housekeeping gene dubbed B-actin. The outcomes of three separate investigations were averaged, and each one was carried out in triplicate.

**Table 1:** The primer sequences of the examined genes along with their GenBank accession numbers.

Gene	Forward primer	Reverse primer	Accession No.
***CyclinE***	CAGAGACAGCTTGGATTTGC	ACTGTCTTTGGTGGAGAA GG	NM_001237.5
***CDK2***	GCTAGCAGACTTTGGACTAGCCAG	AGCTCGGTACCACAGGGTCA	NM_052827.4
***P21***	CGATGGAACTTCGACTTTGTCA	GCACAAGGGTACAAGACAGTG	NM_001374511.1
***Cyclin D1***	TCCAGAGT GATCAAGTGTGA	GATGTCCACGTCCCGCACGT	NM_004994.3
***P27***	GCCCTCCCCAGTCTCTCTTA	TCAAAACTCCCAAGCACCTC	NM_001302510.2
***BCL-2***	CCTGTG GAT GAC TGA GTACC	GAGACA GCC AGG AGAAAT CA	NM_000633.3
***BAX***	GTTTCA TCC AGG ATC GAGCAG	CATCTT CTT CCA GATGGT GA	NM_001291428.2
***Caspase-3***	CAGAACTGGACTGTGGCATTGAG	GGATGAACCAGGAGCCATCCT	NM_004346.4
***CDK4***	CTGGTGTTTGAGCATGTAGACC	AAACTGGCGCATCAGATCCTT	NM_001357943.2

### ELISA testing

The targeted genes’ levels of protein expression were assessed using an ELISA method in HepG2 cells that were recently challenged with green tea extract. In the ELISA process, human Bax ELISA Kit (ab199080), human Bcl-2 Kit (ab272102), human cleaved Caspase-3 Kit (ab220655), human P21 ELISA Kit (ab214658), human Cyclin E1 Kit (ab231929), and human Cyclin D1 ELISA Kit (ab214571) were employed. All of these kits were produced using a single, highly sensitive sandwich enzyme assay that takes 90 minutes to complete. This assay uses antibodies that act as trapping agents linked to the affinity tag and is additionally detected by an exact anti-tag antibody that has been precoated on the testing ELISA plate. The examined extract-containing established HepG2 cells were spun up, and the pellet was then transferred to a 96-well ELISA panel alongside a corresponding quantity of an antibody cocktail solution. The plate was then put away at room temperature for 1 h to permit the antibodies to stick to the sample. After thoroughly rinsing the plate in wash buffer (1x), a tetramethylbenzidine substrate solution was added to each well for ten min. Upon that, the plate was placed in a dim area. Then, immediately following the addition of a stop solution, the intensity at 450 nm was recorded via an automatic microplate reader.

RETRACTED

Similar to the aforementioned, the CDK2 ELISA kit (catalog no. MBS2020144), CDK4 Human ELISA Kit (catalog no. E-EL-H2323, MyBioSource, USA), and P27 Human ELISA Kit (catalog no. E-EL-H0909, MyBioSource, USA) were employed to gauge the amounts of protein expression levels of CDK2, CDK4, and P27, respectively: The 96-well plates contained in these kits, which used sandwich ELISA double-antibody approaches, had already been coated with anti-human CDK2, anti-human CDK4, and anti-human P27 antibodies. The wells were cleaned with washing buffer before adding the test and standard samples (HepG2 cell extract-treated supernatant) and identifying the antibody containing biotin-conjugated antibodies. After that, streptavidin and horseradish peroxidase were applied to the wells, followed by the application of the HRP substrate, which caused the production of a blue hue. The reaction was then halted by adding an acidic solution, which caused the blue color to change to yellow.

### Statistical analysis

All studies were completed three times, and the outcomes are shown as the mean ± standard deviation. All statistical analyses were carried out an employing independent T- test using the SPSS 17.0 software. Statistical significance was assigned to values of p≤ 0.05, p ≤ 0.01, and p ≤ 0.001.

## Results and discussion

### Discovering phytochemical components using GC-MS

A total of 71 compounds were identified by GC-MS analysis; most of them have higher biological activity that may be responsible for the biological effectiveness of the examined green tea extract, with various retention durations indicated in **Fig 1**. The biological activity of these compounds, along with their percentages of the peak area and retention time, is shown in **Table 2**. Thus, the current findings about the anticancer efficacy of the investigated extract of green tea (*Camellia sinensis*) may be attributed to the presence of these components. Most phenolic ingredients, including polyphenols in green tea, have the ability to promote cancer defense in a range of biological operations. Green tea polyphenols are renowned for their powerful antioxidant activities and could be significant in anticancer behavior, protecting pre-malignant cells from DNA damage induced by oxidation **[32]**. Growth arrest and apoptosis can be triggered by other processes besides the antioxidant properties of these phenolic chemicals, which may not be sufficient for their chemopreventive benefits **[33]**.

RETRACTED

**Fig 1:** GC-MS chromatogram of the green tea leaf methanol extract (GTME) for the assessment of phytochemicals. Table 2 lists all the hytochemical TMS derivatives that have been seen in this image.

**Table 2:** Phytochemical components of Camellia sinensis methanolic extract as identified by GC-MS analysis.

Peak No	Retention Time	Area%	Name of the compound	Molecular formula	Molecular weight (g/mol)	Biological activity
**1**	10.2441	0.7119	Acetic acid, 2-[2 [(trimethylsilyl)oxy]ethoxy]-, trimethylsilyl ester	C11H28O4Si3	308.59	Antimicrobial Activity **[34]**
**2**	10.456	0.3113	Silanol, trimethyl-, phosphate (3:1)	C9H27O4PSi3	314.54	Antioxidant, Antibacterial activity **[35]**
**3**	10.874	0.2255	Butanedioic acid, 2TMS derivative	C10H22O4Si2	262.45	Anti-inflammatory, Antimicrobial **[36]**
**4**	11.06	0.268	Glyceric acid, 3TMS derivative	C12H30O4Si3	322.62	Antimicrobial Activity **[37]**
**5**	11.64	0.1019	2-Pentenoic acid, 2-[(trimethylsilyl)oxy]-, trimethylsilyl ester	C11H24O3Si2	260.47	Antibacterial activity **[38]**
**6**	13.088	1.293	Malic Acid, 3TMS derivative	C13H30O5Si3	350.63	Antioxidant, Antibacterial activity **[35]**, Anticarcinogenic activity **[39]**
**7**	13.317	0.1646	meso-Erythritol, 4TMS derivative	C16H42O4Si4	410.84	Sweet antioxidant **[40]**
**8**	13.437	0.085	Diglycolic acid, 2TMS derivative	C8H20O3Si2	220.41	Antioxidant activity**[41]**
**9**	13.689	0.5664	Pyrogallol, 3TMS derivative	C15H30O3Si3	342.65	Antioxidant, Antiseptic, Antibacterial, Anti-tumor Dye **[42,43]**
**10**	13.975	0.8736	Hexanoic acid, 2-hydroxy-2-butyl-, 2 methylphenylhydrazide	C17H28N2O2	292.423	Antifugial activity **[44]**
**11**	14.187	0.1373	o-Coumaric acid, 2TBDMS derivative	C21H36O3Si2	392.7	Anticarcinogenic activity **[45]**
**12**	14.656	0.07	Isoborneol, pentamethyldisilanyl ether	C15H32OSi2	284.58	Antioxidant, Anti-viral Activity **[46]**
**13**	14.948	0.1515	Erythritol, 4TMS derivative	C16H42O4Si4	410.84	Sweet antioxidant **[47]**
**14**	15.062	0.1468	1,2-O-Isopropylidene-.alpha.-D-glucofuranose, 3TMS derivative	C9H16O6	220.22	Antifungal activity **[48]**
**15**	15.274	0.194	L-Rhamnose, 4TMS derivative	C18H44O5Si4	452.88	anti-inflammatory activity **[49]**
**16**	15.485	0.1443	L-Threitol, 4TMS derivative	C16H42O4Si4	410.84	Antibacterial activity **[50]**
**17**	15.731	0.3378	Xylitol, 5TMS derivative	C20H52O5Si5	513.05	Antimicrobial **[51]**
**18**	15.972	0.4722	D-Allose, oxime (isomer 1), 6TMS derivative	C24H61NO6Si6	628.25	Antioxidative Activity **[52]**
**19**	16.081	0.2061	Itaconic acid, 2TMS derivative	C11H22O4Si2	274.46	Anti-inflammation activity **[53]**
**20**	16.367	3.1304	Fructofuranoside, methyl 1,3,4,6-tetrakis-O-(trimethylsilyl)-,.alpha.-D-	C19H46O6Si4	482.9	Anti-Oxidant activity **[54]**
**21**	16.767	7.2397	6-Hydroxyflavone-beta-D-glucoside, tetra(trimethylsilyl)-	C33H52O8Si4	689.1	Anticancer and antioxidant **[55]**
**22**	17.128	3.5932	Pyrimidin-2-amine, 4-methyl-6-(2-pyridylthio)-	C10H10	218.27	Antifungal Activity **[56]**
**23**	17.231	3.7531	Quininic acid (5TMS)	C22H52O6Si5	553.1	Antibacterial activity **[57]**
**24**	17.425	3.2087	2-Butenoic acid, 2-[(tert-butyldimethylsilyl)oxy]-, tert-butyldimethylsilyl ester	C17H36O3Si2	344.64	antioxidant, anti-inflammatory activity **[58]**
**25**	17.597	2.8917	2-Carboxycinnamic acid	C10H8O4	192.17	Antioxidant **[59]**
**26**	17.803	3.1585	Deoxyglucose, 4TMS derivative	C18H44O5Si4	452.88	Anticancer activity **[60]**
**27**	17.992	3.7033	D-Mannitol, 6TMS derivative	C24H62O6Si6	615.25	Anti-bacterial Activity [61]
**28**	18.129	0.8268	Caffeine	C8H10N4O2	194.19	Anticancer activity **[62]**, antioxidant, anti-inflammatory **[63]**
**29**	18.301	2.2683	Gallic acid, 4TMS derivative	C19H38O5Si4	458.84	Antioxidant **[64]**, antimicrobial **[65]**, antifungal **[66]**, anticancer **[67]**
**30**	18.449	1.2158	Arabinofuranose, 1,2,3,5-tetrakis-O-(trimethylsilyl)-	C17H42O5Si4	438.9	Antibacterial Activity **[68]**
**31**	18.695	3.0842	Glycine, 2TBDMS derivative	C14H33NO2Si2	303.58	Antioxidant and Antimicrobial Activity **[69]**
**32**	18.936	0.9875	L-(+)-Tartaric acid, 4TMS derivative	C16H38O6Si4	438.81	Antimicrobial, Antioxidant activity **[70]**
**33**	19.279	0.192	Palmitic Acid, TMS derivative	C19H40O2Si	328.60	anticancer, anti-inflammatory activity **[71]**
**34**	19.823	0.8974	Levoglucosan, 3TMS derivative	C15H34O5Si3	378.68	Anticancer and antitumor activity **[72]**
**35**	19.983	0.1959	Myo-Inositol, 6TMS derivative	C24H60O6Si6	613.24	Anticancer activity **[73]**
**36**	21.144	0.4077	D-(+)-Galactopyranose, 5TMS derivative	C21H52O6Si5	541.06	Antibacterial activity **[74]**
**37**	21.402	0.1416	6-Hydroxyfavone-beta-D-glucoside, tetra(trimethylsilyl)-	C_33_H_52_O_8_Si_4_	689.1	Anticancer and antioxidant **[75]**
**38**	21.562	0.0808	D-(+)-Galacturonic acid, 5TMS derivative	C21H50O7Si5	555.04	antioxidative and anticancer effects **[76]**
**39**	21.877	1.6205	Maltitol, nonakis(trimethylsilyl) ether	C39H96O11Si9	993.94	Antibacterial activity **[77]**
**40**	22.203	0.3366	Oxalic acid, 2TMS derivative	C8H18O4Si2	234.39	No reported activity
**41**	22.363	0.256	Molybdenum, tricarbonyl[(1,2,3,4,5,6-.eta.)-1,4-dimethylbenzene]-	C11H10MoO3	286.14	Anticancer and antidiabetic Activity **[78]**
**42**	22.569	0.2573	D-Ribose, 4TMS derivative	C5H10O5	150.12	antiviral, anti-tubercular and anti-inflammatory activities **[79]**
**43**	22.684	0.496	D-Glucuronic acid, 2,3,4,5-tetrakis-O-(trimethylsilyl)-, trimethylsilyl ester	C21H50O7Si5	555.04	detoxification and protection of the liver **[80]**
**44**	22.975	0.3299	Glycerol, 3TMS derivative	C12H32O3Si3	308.63	antimicrobial activities **[81]**
**45**	23.267	0.831	Salicylic acid, 2TMS derivative	C13H22O3Si2	282.48	Antioxidant activity **[82]**
**46**	23.445	0.4667	D-(+)-Xylose, tetrakis(trimethylsilyl) ether, methyloxime (syn)	C18H45NO5Si4	467.89	Antibacterial **[83]**
**47**	23.668	3.0311	Sucrose, 8TMS derivative	C36H86O11Si8	919.74	Antibacterial **[83]**
**48**	23.851	2.7647	Lactulose,octakis(trimethylsilyl) ether, methyloxime (isomer 2)	C37H89NO11Si8	948.79	Prebiotic activity **[84]**, anti tubulointerstitial fibrosis **[85]**
**49**	24.04	3.8229	D-(-)-Ribofuranose, tetrakis(trimethylsilyl) ether	C17H42O5Si4	438.85	antiviral, anti-tubercular and anti-inflammatory activities **[79]**
**50**	24.246	5.1177	Xylonic acid, 2,3,4-tris-O-(trimethylsilyl)-,.delta.-lactone, D-	C14H32O5Si3	364.65	antiviral and antimicrobial activity **[86]**
**51**	24.412	2.956	Thymol-.beta.-d-glucopyranoside, tetrakis(O-trimethylsilyl)-	C28H56O6Si4	601.1	Antibacterial **[87]**
**52**	24.583	1.59	Methyl.beta.-Arabinofuranoside, 3TMS derivative	C15H36O5Si3	380.2	Antioxidant Activity **[88]**
**53**	24.732	1.8818	Uridine, 3TMS derivative	C18H36N2O6Si3	460.74	Antimicrobial, anticancer activity **[39]**
**54**	24.921	2.8263	D-Arabinopyranose, 4TMS derivative (isomer 2)	C17H42O5Si4	438.85	Antioxidant Activity **[88]**
**55**	25.201	1.3047	2-O-Glycerol-.alpha.-d-galactopyranoside, hexa-TMS	C27H66O8Si6	687.32	antimicrobial activities **[81]**
**56**	25.39	5.1465	D-Xylopyranose, 4TMS derivative	C17H42O5Si4	438.85	Antibacterial and antimicrobial activity **[86]**
**57**	25.705	2.5646	alpha.-D-Glucopyranose, 5TMS derivative	C21H52O6Si5	541.06	antifungal activity antimalaria activity **[89]**
**58**	25.894	0.895	2,5-Dihydroxybenzoic acid, 3TMS derivative	C16H30O4Si3	370.66	Antipyretic analgesic, antirheumatism, and antimicrobial activity **[90]**
**59**	26.031	2.136	1H-Indole, 3-phenyl-2-(3’-phenyl-1H-indol-2’-yl)-	C28H20N2	384.5	Antioxidant activity and anticancer activity **[91]**
**60**	26.266	0.9705	Caffeic acid, 3TMS derivative	C18H32O4Si3	396.70	Antioxidant and anticarcinogenic **[92]**
**61**	26.529	1.3675	Phenanthrene, 4-methyl-	C15H12	192.25	Antitumor and antimicrobial **[93]**
**62**	26.706	0.7119	alpha.-D-Lactose, 8TMS derivative	C36H86O11Si8	919.74	Antibacterial **[83]**
**63**	27.05	0.9501	Cycloheptasiloxane, tetradecamethyl-	C14H42O7Si7	519.07	antibacterial and antioxidant activity **[94]**
**64**	27.204	0.6473	Serine, 3TMS derivative	C12H31NO3Si3	321.63	No reported activity
**65**	27.616	0.9969	Maltose, octakis(trimethylsilyl) ether, methyloxime (isomer 2)	C37H89NO11Si8	948.78	Antibacterial **[95]**
**66**	27.782	0.4683	3-.alpha.-Mannobiose, octakis(trimethylsilyl) ether (isomer 1)	C36H86O11Si8	919.745	No reported activity
67	28.017	1.2909	Arabinose, 4TMS derivative	C17H42O5Si4	438.85	Antibacterial **[96]**
**68**	28.429	2.177	.beta.-L-Arabinopyranose, 4TMS derivative	C17H42O5Si4	438.85	Antioxidant Activity **[88]**
**69**	29.121	0.1613	2-Pentenedioic acid, 2-[(trimethylsilyl)oxy]-, bis(trimethylsilyl) ester	C14H30O5Si3	362.64	Anti-inflammatory **[97]**
**70**	29.527	1.9118	Benzoic acid, 3-amino-5-hydroxy-tris(trimethylsilyl) derivative	C16H31NO3Si3	369.68	No reported activity
**71**	30.528	0.2771	Protocatechoic acid, 3TMS derivative	C16H30O4Si3	370.66	antioxidative and anti-inflammatory activity **[98]**

RETRACTED

### Estimation of total phenolic, flavonoids and tannins

Phenolic and flavonoid components in medicinal herbs are the main sources of antioxidants. Numerous plant secondary metabolites have been shown to possess pharmacological properties including antioxidant, antifungal, anticancer, and antibacterial properties, as well as to be physiologically active compounds **[99]**. They may also aid in the prevention of chronic diseases. GTME’s flavonoids and polyphenols can protect cells from oxidative stress, which reduces the likelihood that oxidative stress will lead to the development of cancer **[100]**. The current acquired results demonstrated that the total phenolic, flavonoid, and tannin content in the examined GTME was 128.8±3.12 mg of GAE, 83.74±2.61 mg of QE, and 11.66±1.23 mg of TAE per g of the GTME, respectively, based on the standard calibration plots for GAE, QE, and TAE. Phenolic compounds have the ability to scavenge singlet oxygen, free radicals, and superoxide radicals because of their redox properties **[101]**. Because hydroxyl groups replace the aromatic ring in polyphenolic compounds, they have the ability to scavenge radicals **[102]**. The antioxidant qualities of flavonoids, which are plant secondary metabolites, including flavones, flavanols, and tannins, depend on the presence of free OH groups, especially 3-OH. Furthermore, other studies have shown that flavonoids from plants function as antioxidants in vivo as well as *in vitro* **[103,104]**. Furthermore, earlier studies demonstrated that green leaf methanol extract included notable concentrations of phenols, tannins, and flavonoids **[105]**.

### Efficiency of GTME on proliferation of HepG2 cells

#### MTT cytotoxicity assay

It was mentioned that the use of natural phytochemicals in cancer chemoprevention is an increasingly popular approach to preventing, slowing down, halting, and treating malignant tumors **[25]**. Thus, MTT investigations were performed to figure out the adverse impacts of the investigated GTME on the proliferation of HepG2 cells. By incorporating the MTT test, the findings demonstrated that the proportion of viable HepG2 cells drastically decreased in a concentration-related manner after being exposed to the analyzed extract for 24 h **(Fig 2A)**. This discovery might highlight the extract’s potential anticancer properties, which can be determined by its lower IC_50_ dose (27.3 µg/ml). This was calculated based on the link within the extract dose and how it affected cell life expectancy. Likewise, it has been verified that green tea plant extract suppresses the development of numerous cancer cell lines, occasionally due to its antioxidant qualities **[106]**. Also, methanol green tea extract has been shown to be effective in inhibiting the growth of human cervical cancer cells **[19]** and renal carcinoma cells **[20]**. Curcumin, an anticancer drug, was shown in earlier research to have an inhibitory effect on HepG2 cells after a 24-hour treatment period (IC50 value: 48.70 µg/ml) **[107]**.

**Fig 2:** The cytotoxicity of HepG2 (a) and the viability of WI-38 cells (b) after 24 h of incubation against various doses of green tea methanol extract (GTME). The values are compared to the control (untreated cells), * *p* < 0.05.

Results from culturing human lung normal cells, WI-38 cells, with GTME at concentrations ranging from 31.25 to 500 µg/ml are presented in **Fig 2B**, which reveal a significantly increased percentage of cell viability with an IC_50_ concentration equal to 2757.2 µg/ml. These results showed that the GTME was toxic to cancer cells while being non-toxic and biocompatible with healthy tissue. Previous research **[108]** has demonstrated that the IC_50_ concentration of curcumin against non-cancerous WI-38 cells was 6.56 µg/ml, suggesting that the produced GTME is more safe than the anticancer medicine curcumin.

RETRACTED

#### Estimation of HepG2 cells’ apoptosis generation

The evaluated GTME’s ability to induce apoptosis in HepG2 cells was assessed using a number of assays involving annexin V/PI, AO/EB, and comet. Beginning with **Fig 3**, displaying the flow cytometry-derived annexin V/PI for the extract-treated cells contrasted with untreated ones, it might be seen that, compared to the control cells, the extract-treated HepG2 cells possessed a larger proportion of early and late apoptotic cells. Previous research has shown that curcumin, an anticancer drug, dramatically boosted HepG2 cell death in a dose- and time-dependent manner **[109].**

**Fig 3:** Using flow cytometry, the apoptotic pattern of HepG2 cells was assessed, displaying Q1 (An−, PI+) % of necrotic cells, Q2 (An+, PI+) % of late apoptotic cells, Q3 (An−, PI−) % of viable cells, and Q4 (An+, PI−) % of early apoptotic cells for treated GTME cells with an IC50 dose (27.3µg/ml) of GTME (b) in comparison to untreated HepG2 cells (a).

In addition, a quantitative AO/EB protocol that is in particular made for nuclear labeling of apoptotic cells was applied to compute the percentages of apoptotic cells in HepG2 cells treated with green tea extract and to assess how apoptotic cells’ altered nuclear morphology. As indicated by **Fig 4**, green, yellow-green, and orange hues were produced in the extract-treated HepG2 cells **(Fig 4B)**, suggesting the existence of viable, early, and late apoptotic cells. While the green viable control cells **(Fig 4A)** did not show any discernible apoptosis, in contrast to control cells (9.5± 0.58), the percent of apoptotic cells was significantly greater in treated cells (90.5± 2.65). According to prior studies, Epigallocatechin-3-gallate has been shown to trigger apoptosis in a variety of human cancer cells, including those of the pancreas **[110]** and the colon **[111]**, via modulating apoptosis related proteins. Additionally, prior studies employing the AO/EB test showed that curcumin induced morphological and staining alterations in treated HepG2 cells were suggestive of both early and late apoptosis **[112]**. The AO/EB test for the extract’s consequence on healthy WI-38 cells revealed, as shown in **Fig 4C and 4D**, that the GTME-treated WI-38 cells had a shade of green that was comparable to the green color seen in untreated cells and lacked any obvious symptoms of apoptosis.

RETRACTED

**Fig 4:** Using fluorescence microscopy and AO/EB labelling, the nuclear morphological alterations in treated HepG2 cells with an IC_50_ dose (27.3µg/ml) of GTME (b) in comparison to untreated HepG2 cells (a) and also GTME treated normal WI-38 cells (d) in comparison to untreated WI-38 cells (c) have been observed. All images are at 40X magnification.

The comet strategy is also used to detect DNA damage brought on by treated cells starting to go into apoptosis. Moreover, fluorescent microscopy imagery **(Fig 5)** indicated that treated cells **(Fig 5B)** had a comet-like structure with an increment in the tail length, indicating that a disproportionate buildup of DNA in the tail perhaps caused the nuclear density to decline, in contradiction to the control cells **(Fig 5A)**, which maintained their fundamental nuclear structure. Caspase3 (activated caspase-3), as stated earlier, is essential for the apoptosis-mediated cell death process, which causes DNA fragmentation and nuclear condensation **[113]**. According to **Table 3**, the OTM of the GTME-treated and untreated cells was significantly different. Previous investigations have indicated that large doses of the anticancer drug curcumin can cause damage to the nuclear DNA of HepG2 cells **[114]**.

**Fig 5:** Fluorescence microscopy of the comet nucleus in treated HepG2 cells with an IC_50_ dose (27.3µg/ml) of GTME (b) in comparison to an intact nucleus in untreated HepG2 control cells (a) and in treated WI-38 cells with GTME (d) in comparison to untreated WI-38 control cells (c). All images are at 40X magnification.

**Table 3:** The comet parameters in HepG2 cells treated with GTME and control untreated HepG2 cells, as well as in WI-38 cells treated with GTME and control untreated WI-38 cells, were determined using the comet assay.

The tested cells	Tail length (px)	%DNA in tail	Tail moment	Olive tail moment
**Control HepG2 cells**	8.58 ± 1.35	5.06 ± 0.31	0.41 ± 0.01	0.54 ± 0.02
**Treated HepG2 cells with the green tea extract (GTME)**	9.56 ± 0.52	13.83 ± 0.52 ^**a**^	1.34 ± 0.04 ^**a**^	1.89 ± 0.04 ^**a**^
**Control WI-38 cells**	10.42 ± 1.63	7.40 ± 2.21	0.74 ± 0.04	1.11 ± 0.03
**Treated WI-38 cells with the green tea extract (GTME)**	9.56 ± 2.62	7.65 ± 1.83	0.78 ± 0.02	1.13 ± 0.02

Data from three separate tests are presented as the mean ± standard deviation. Statistically significant (p < 0.05) differences are shown by lowercase letters. ^**a**^ (p < 0.05) with respect to control HepG2 cells.

In an effort to confirm caspase-3’s essential role in DNA fragmentation and the execution of apoptosis in treated HepG2 cells, the extract’s impact on Caspase-3 expression was assessed. The outcomes demonstrated that the treated cells expressed more caspase-3 than the control cells. Previous studies have also shown that DNA fragmentation is a hallmark of apoptosis produced by green tea polyphenols in MCF-7 cells **[115]**. Additionally, the comet analysis results for the impact of the GTME on the DNA of normal WI-38 cells are consistent with the OTM values of the control cells and the cells treated with the tested extract, which were not significantly opposed to one another **(Table 3)**. The comet fluorescence results in the extract-treated WI-38 cells, which showed an undamaged, intact nucleus, provided additional proof that the extract had no genotoxic effects on healthy, alive tissues. **(Fig 5D)** is the same as the healthy nucleus of control cells without any effect on DNA **(Fig 5C)**.

RETRACTED

#### Cell cycle analysis

One of the primary strategies for preventing the spread of cancer is to inhibit the cell cycle’s progression **[116]**. Therefore, it was possible to examine the data using flow cytometry to determine how the investigated extract affected the regulation of the HepG2 cell cycle phases. **Fig 6A–6C**. The control cells did not exhibit any apoptosis-related symptoms, as shown in **Fig 6A**, while in treated HepG2 cells, the green tea extract resulted in a significantly larger percentage of apoptotic cells in the sub-G1 phase with a pausing in the G1 phase **(Fig 6B)**, demonstrating that it causes apoptosis. The ratios of the cell population throughout each stage of the HepG2 cell cycle are shown in a typical histogram that compares control cells with cells treated with the extract. **(Fig 6C)**. Likewise, previous studies demonstrated that the appositive anticancer medication curcumin caused G1 phase stopping in HepG2 treated cells **[117]**.

**Fig 6:** Flow cytometric examination of the distribution of the cell cycle at various stages in control HepG2 cells (a) and in HepG2 cells that had been treated with an IC_50_ dose (27.3 µg/ml) of green tea extract (GTME) (b). An illustration of a histogram that displays the proportions of cells in each stage of the cell cycle in untreated and GTME-treated cells (c). Statistically significant (p < 0.05) differences are shown by lowercase letters. ^**a**^ (p < 0.05) with respect to control cells.

Green tea polyphenols have been demonstrated to elicit cell cycle arrest in MCF-7 breast cancer cells at the G1/S and G2/M transitions **[115]**. Also, earlier studies have revealed that the polyphenolic substance found in green tea, called epigallocatechin-3-gallate, can induce cell cycle halt at the G1 phase in several human cancer cells, including pancreatic **[110]**, head and neck squamous carcinoma **[118],** and colon **[119],** via modulating proteins that control the G1 phase of the cell cycle. Numerous signaling molecules and checkpoints (CDKs) that control cell division mediate cell proliferation. On the one hand, the combination of cyclins (D and E) and cyclin-dependent kinases (CDK4, CDK6, and CDK2) positively controls cell cycle progression. which releases the E2F transcription factors and phosphorylates the retinoblastoma tumor suppressor (pRb) protein to allow cells to move from the G1 phase to the S phase. On the other hand, the kinase inhibitor proteins p21, p27, and p57 bind to the cyclin D/CDKs (4 or 6) complex or the cyclin E/CDK2 complex and prevent the G1/S transition **[120]**. Therefore, in the current investigation, QRT-PCR and ELISA were used to ascertain the expression levels of P21, P27, CDK2, CDK4, Cyclin D1, and Cyclin E in the extract-treated cells. The data that was obtained demonstrated that the extract enhanced P21 and P27 expression while decreasing CDK2, CDK4, Cyclin D1, and Cyclin E expression in treated HepG2 cells, proving their roles in halting the treated HepG2 cell at the S phase.

RETRACTED

#### Effect of GTME on ROS induction in HepG2 cells

Due to their heightened metabolic activity, most cancerous cells have high quantities of ROS, and these ROS have specific functions in the development of cancer cells such as angiogenesis, cell cycle progression, cell survival, and cell proliferation **[121]**. Earlier research has shown that ROS downregulation causes apoptosis **[122]**, suggesting that ROS inhibition could be an effective cancer treatment **[123]**. In the obtained finding, the GTME significantly reduced ROS levels in the treated cells when compared to control cells (p < 0.05), as shown in **Fig 7**. This suggests that the triggering of apoptosis in cells treated with green tea extract may be connected to the extract’s capacity to lower ROS levels. Similar findings were made by prior research, which showed that the methanol extract of stevia and Smallanthus sonchifolius leaves decreased ROS in SKVO3 and HepG2 cells **[25,124]**, respectively, as compared to control cells. This finally resulted in apoptosis. However, previous research has shown that the anticancer drug curcumin dramatically raised the levels of ROS inside HepG2 cells, causing apoptosis **[125].**

**Fig 7:** The quantity of reactive oxygen species (ROS) present in the HepG2 cells after treatment with an IC_50_ dose (27.3 µg/ml) of green tea extract (GTME) when compared to untreated cells. Statistically significant (p < 0.05) differences are shown by lowercase letters. ^**a**^ (p < 0.05) with respect to control cells.

RETRACTED

#### Quantification analysis using qRT-PCR and ELISA assays

Proapoptotic controllers (BAX, BAK, and BAD) and antiapoptotic controllers (BCL-2 and BCL-XL) are all members of the BCL-2 protein family, which regulates apoptosis **[126]**. Furthermore, mitochondrial permeabilization brought on by BAX overexpression increases Cytochrome c release into the cytoplasm, which in turn activates *Caspase-3* **[127]**. In this way, caspase3 activation triggers DNA damage, apoptosis, and a decrease in BCL2 gene expression **[128]**. Additionally, the kinase inhibitor proteins P21, P27, and P57 bind to the cyclin D/CDKs (4 or 6) complex or the cyclin E/CDK2 complex and prevent the G1/S transition **[120]**. So, in the present investigation, the effects of green tea extract on the levels of mRNA expression for genes associated with apoptosis (*BCL2*, *BAX*, *and Caspase-3*) and G1-phase cell cycle arrest (*P21*, *P27*, *CDK2*, *CDK4*, *Cyclin E*, *and Cyclin D1*) were assessed. Expressed levels of *BAX* and *Caspase-3* were found to be significantly increased, while *BCL-2* expression was found to be significantly decreased in the GTME-treated cells compared to the control cells, p < 0.05 **(Fig 8)**. These results suggest that the GTME-treated HepG2 cells’ induction of apoptosis may have included the mitochondrial pathway. Prior studies have shown that the appositive anticancer medication curcumin exhibited a similar impact on the proteins implicated in programmed cell death in HepG2 cells. The apoptotic proteins caspase-3 and Bax were upregulated in HepG2 cells treated with curcumin, whereas the anti-apoptotic protein Bcl-2 was downregulated, causing induction of the mitochondrial apoptosis pathway **[129]**. In addition, the obtained green tea extract markedly elevated the expression levels of P21 and P27 genes while significantly lowering the expression of CDK2, CDK4, Cyclin E, and Cyclin D1, p < 0.05 (**Fig 8**), indicating that the GTME produced G1 arrest in the treated HepG2 cells by controlling proteins associated with the G1/S phase.

**Fig 8:** The effects of the green tea extract (GTME) at the IC_50_ dose (27.3 µg/ml) on the expression levels of *Bax*, *P21*, *Caspase-3*, *P27*, *Cyclin E*, *CDK2*, *Bcl-2*, *CDK4*, *and Cyclin D1* in HepG2-treated cells were compared to control cells using qRT-PCR. Statistically significant (p < 0.05) differences are shown by lowercase letters. ^**a**^ (p < 0.05) with respect to control cells.

In an effort to verify the levels of mRNA expression of all evaluated genes, the proteins that these genes express were tested in the GTME-treated cells using the ELISA test. The findings are displayed in **Fig 9**, which confirms that the treated cells exhibit significant elevated levels of the proteins Bax, P27, P21, and cleaved Caspase-3, while exhibit significant downregulated levels of CDK2, CDK4, Cyclin E, Cyclin D1, and Bcl-2 as compared to untreated cells. According to these results, which were in line with those of the aforementioned qRT-PCR, the tested green tea extract significantly raised the changes in apoptosis and G1-phase cell cycle arresting proteins within HepG2- treated cells as compared to the control cells.

RETRACTED

**Fig 9:** The effect of the IC_50_ dose (27.3µg/ml) of green tea extract (GTME) on the protein content of Cyclin E, Cyclin D1, Bcl-2, CDk2, CDK4, Bax, cleaved Caspase-3, P27, and P21 in HepG2-treated cells compared to that of control cells using the ELISA method. Statistically significant (p < 0.05) differences are shown by lowercase letters. ^**a**^ (p < 0.05) with respect to control cells.

## Conclusion

In the present investigation, a connection was established among the bioactive phytochemical components (antioxidant and anticancer ingredients) present in the generated hydromethanolic extract of green tea leaves (GTME) and the extract’s powerful outcomes on the viability of the tested HepG2 cancer cells. With a substantial IC_50_ value of 27.3µg/ml of the tested GTME, it had an improved effect on HepG2 cells in terms of inducing apoptosis, preventing the cell cycle at the G1 phase with a higher proportion of apoptotic cells in sub-G1, and lowering ROS levels in comparison to control cells. Furthermore, the extract affected proteins involved in apoptosis and G1 cell cycle arrest in HepG2- treated cells as compared to control cells. Green tea leaf extract (GTME) shows promise as a natural therapy for human liver cancer, as suggested by these results. *In vivo* studies using animal models are crucial for providing evidence for these findings.

## Abbreviations

MTT 3: (4,5-Dimethylthiazol-2-yl)-2,5-diphenyltetrazolium bromide
IC_50_: Half maximal inhibitory concentration
ELISA: Enzyme-linked immunosorbent assay
Bax: Bcl-2 Associated X-protein
Bcl-2: B-cell lymphoma 2
CDK2: Cyclin dependent kinase 2
CDK4: Cyclin-Dependent Kinase 4
